The article "Green Innovation and Enterprise Sustainable Development Performance Based on the SBM-DEA Model" was retracted in 2023. Reasons: unreliable results or conclusions; concerns about the data; concerns about the peer review; concerns about the citations.

# Green Innovation and Enterprise Sustainable Development Performance Based on the SBM-DEA Model

**DOI:** 10.1155/2022/3127899

**Published:** 2022-08-30

**Authors:** Ning Han, Feng Li, Jing Long, Jing Liu, Qianyun Li

**Affiliations:** Chengdu Jincheng College, Chengdu 610000, Sichuan, China

## Abstract

Since the introduction of a low-carbon economy, corporate performance is no longer limited to the evaluation of internal economic benefits but has become the performance of corporate sustainable development, adding environmental and social factors. Now, the whole world is paying attention to low consumption and low emission. As the main economic pillar of society, the enterprise undertakes the biggest low-carbon task. In order to develop the economy in the longer term and meet the needs of society, enterprises must combine green innovation to evaluate the performance of sustainable development. However, because the previous model's analysis of performance will produce distortion effects, the data error is also relatively large. Therefore, in order to solve these problems and make performance analysis more realistic, this paper deeply discusses the issue of green innovation and enterprise sustainable development performance. Using the method of the SBM-DEA model, it analyzes the performance comparison of enterprises without and with the expected output and conducts a comparison experiment. The result shows that in 2017, the efficiency of company A without unexpected output was 0.6943. The efficiency with undesired output is 0.6643. In 2018, the efficiency of the enterprise without undesired output is 1, and the efficiency with undesired output is 1. After applying the model, it is obvious that the efficiency of computing performance has been greatly improved. Therefore, in order to better study the sustainable development performance of enterprises, the SBM-DEA model should be focused on.

## 1. Introduction

China's economy continues to achieve new high-speed growth, but the price of this growth is the destruction of the natural environment and the consumption of natural energy. In the process of economic development, human beings have produced too many sources of pollution, and these pollutants have squeezed the bearing capacity of the Earth's environment. It leads to extreme ecological imbalance and global warming; some harmful substances affect the health of many people; and natural resources are gradually depleted. This is undoubtedly another warning from the Earth to mankind, there is only one Earth, and these injuries are of a global nature. Through relevant surveys, it can be found that the pollutants emitted by enterprises are the largest. Therefore, enterprises should undertake this social responsibility, formulate green innovation strategies, and attach importance to the implementation of the concept of sustainable development. By deepening the concept of green development, innovating technological models, and improving corporate performance, a positive corporate social image should be created. At present, many scholars have studied the topic of green innovation and enterprise sustainable development performance, but there are relatively few studies using the SBM-DEA model. The SBM-DEA model is an efficiency evaluation method. It can solve the slack problem of input and output and reduce the impact of undesired output on efficiency measurement. If the model is applied to the analysis of green innovation and enterprise sustainable development performance, it is believed that it can get good results.

The implementation of enterprise green innovation strategy is to make enterprises pay more attention to green management, reduce waste of resources, and enhance the thinking of caring for the environment. Many scholars have also done research on green innovation and corporate sustainability performance. Guan [1] studied the innovation management performance evaluation model of papermaking enterprises based on organizational shared thinking and constructed a management structure model [1]. However, he did not explain much about the concept of organizational mind sharing in the text. Randeree and Ahmend [2] studied the case of Masdar City's urban sustainable development strategy and used it to verify the social sustainable development effect of eco-city [2]. The analytical description they develop in the text lacks a conclusion. Zhang and Lin [3] used quantitative analysis methods to study the high-quality development of the urban economy from multiple aspects and found that innovative green strategies are very suitable [3]. However, they did not make a comparison of urban and rural incomes in the article. He and Shi [4] discussed the impact of environmental regulation on the performance of exploratory innovation, developmental innovation, and green innovation of enterprises [4]. The model they choose in the text is not very suitable.

After analyzing the research results of other scholars, Singh et al. [5] studied the relationship between green innovation strategy and corporate performance and found a positive correlation [5]. But the experiments they conducted in the paper did not take into account the existence of possible influencing factors. Yiyun [6] used the spatial measurement method to test the green innovation ability and performance of enterprises, and the result showed that the competitive relationship can help enterprises develop better [6]. But none of the data he used in the text is up-to-date. Zhang [7] studied the innovation and green development of many enterprises and found that the development of a green economy can effectively improve the performance of enterprises [7]. But he did not describe the before and after comparison of enterprise performance in the article.

The SBM-DEA model has a very wide range of applications, and it has many advantages. It has very good advantages in simplifying the algorithm and reducing errors. The innovation of this paper is to use a novel method, the SBM-DEA model, to study green innovation and enterprise sustainable development performance. In the research process, relevant data and analysis are used in a convenient way to provide support for future green innovation and enterprise sustainable development performance analysis.

## 2. Method of Green Innovation and Enterprise Sustainable Development Performance

### 2.1. Green Innovation

Green innovation is to make full use of human and financial resources and knowledge under the premise of protecting the amount of energy and the natural environment to achieve economic, environmental, and social gains. The process of achieving this is green innovation [8]. Green innovation also includes a lot of content, as shown in Figure 1.

From the information in Figure 1, the difference between green innovation and the innovation advocated before is still very obvious [9]. Green innovation needs to consider the issue of protecting the environment. Its purpose is not only to improve the economic level of enterprises but also to ensure ecological balance and coordinate the conflict between the environment and economic development to ensure the sustainability of enterprise development. Green innovation is not just about technological innovation, not just to meet the needs of the market; the government will also provide corresponding policies to promote its changes. Therefore, green technology, market demand, and government policy are its three aspects, and these three aspects also promote its progress. We can find that green technology has the greatest effect on it. At present, the country is vigorously carrying out the implementation and research and development of green technology, combining green technology with the Internet to improve the labor force. It reduces high energy consumption, reduces pollutant emissions, and effectively improves the natural environment. In fact, the main purpose of designing green innovation activities is to protect ecological resources, study the transformation of different substances, and let new energy technologies replace high energy consumption methods. This makes economic development green and harmonious. Through its construction of a green and economical society, the ecological balance has been maintained. Therefore, in general, green innovation is to make economic development and ecological balance on the same front, check and balance each other, and advance together, thereby promoting the generation of new technologies and reducing energy consumption and pollutant emissions.

The concept of green innovation is given above. Below, we summarize the indicators of green innovation [10], as shown in Figure 2.

Information can be obtained from Figure 2, which has a total of six indicators [11]. The first indicator is the innovation object, mainly about products, services, and production methods. Product innovation is to make the product more green concept and make it circulate in the market, which brings people a better sense of experience. The innovation of services is to integrate the current low-carbon requirements, so as to eliminate waste and increase the burden on the Earth. In the process of service, users can also experience the wind of green saving. The innovation of production methods is the most important part because, according to our investigation, most of the production methods in the country currently bring many pollutants. This has a great impact on the ecological environment. There is only one Earth, and environmental pollution is of a global nature. Therefore, it is necessary to change production methods and optimize innovation methods so that it can implement the concept of green and low-carbon. The second indicator is market positioning, which mainly refers to the need to meet the needs of customers and the competitive environment of the market. Due to the introduction of low-carbon policies, people's awareness of environmental protection has been strengthened. The needs of customers are also gradually linked to green and low-carbon, so the current market positioning is also to be green, low-carbon, and environmentally friendly. The competitive environment of the market should also be positive, and the concept of green innovation should be implemented. The third indicator is environmental benefits, and the environment is the most important indicator here. The introduction of green innovation is to improve the ecological environment and reduce the harm caused to the environment when developing the economy, hoping that the economy can move forward in harmony with the environment. The fourth indicator is the effect stage. What it means is to include the present and the future, to apply this green principle all the time. The fifth indicator is innovation motivation. There is a motivation to do everything, and innovation also has a motivation. It is mainly to minimize the damage to the environment. The sixth indicator is the level of innovation, and the level of innovation is also different, and different standards can be completed from different levels of enterprises, departments, and individuals [12].

### 2.2. Sustainable Development

Sustainable development is a long-term economic growth model [13]. Its ideal state is to meet the needs of current people without affecting the continued development of future generations. It is actually the thought that people get after realizing the seriousness and then reflecting on the ecological destruction [14]. It is a concept that is being promoted all over the world now. It has several basic principles, which can be seen in Figure 3.

Information can be obtained from Figure 3, which has a total of six basic principles [15]. The first principle is the principle of fairness, which mainly means fairness when everything chooses a chance. Creatures in the Earth's ecological cycle predate human beings' possible existence. Our uncontrolled and excessive consumption of the Earth's resources has caused irreparable damage to the space environment in which they live [16, 17]. It is not fair to them. There is also the fairness of predecessors and future generations, and the Earth's resources are not inexhaustible. It is quantitative. If predecessors consume resources excessively, future generations will not get any resources and will clean up the mess left by predecessors. This is not fair to posterity [18]. The second principle is the principle of sustainability, which is the most important part of the six principles. What it means is to emphasize the continuous use of resources and to maintain normal productivity even if the ecology is disturbed by the outside world. To rationally develop and utilize natural resources, the population size should be controlled as much as possible, and the relationship between the economy and the natural environment should be coordinated. The third principle is the principle of harmony, which is an explanation of sustainable development. It means to pay attention to the peaceful coexistence between man and nature [19]. It is hoped that human beings can abide by the laws of nature and treat the natural environment sincerely so that people and nature can interact and make progress together. The fourth principle is demand. It advocates meeting the needs of all people, not selling people's needs as commodities, and creating a vision of a better life. The fifth principle is the principle of efficiency. It means that efficiency is not measured in terms of productivity but in terms of people's actual satisfaction. The sixth principle is stepwise [20]. It mainly says that because of the progress of society, people's requirements will be higher, so future development will change from a low level to a high level.

It also has several connotations, as shown in Figure 4:

Information can be obtained from Figure 4, and its connotation has four points [21]. The first point is to highlight new development themes. It does not blindly pursue economic growth; it considers various factors, such as society, culture, technology, environment, and so on. It pays attention to the rights that people have in common, and countries at any stage have the same right to development. No one can take away this right. The second point is the sustainability of development, and the starting point for this is the ecological environment. It advocates that when human beings develop society and economy, they should consider reducing their impact on the environment. We cannot just focus on production without restraint, without considering the issue of protecting the environment. Once the natural environment can no longer bear it, human beings will suffer a backlash. The third connotation is the fairness of human-human relations. It means that even if the current generation cannot plant trees and let others enjoy the shade, they should not use up resources prematurely so that future generations have no resources to use. Opportunities between people should be equal. Whether it is predecessors or future generations, everyone should get the same resources. The development of the previous generation should not harm the interests of the next generation. Therefore, we must pay attention to sustainable development so that resources can be used effectively and long-term development. The fourth point is the harmonious coexistence of man and nature [22]. People need to know that there is only one Earth. If the ecological balance of the Earth is destroyed by human beings, then only the extinction of human beings will be greeted. Therefore, human beings must establish a new green concept, learn to respect nature, protect nature, and achieve the realm of peaceful coexistence between man and nature. People do not just ask for nature; we can also give back to nature, invent more new energy technologies, replace high energy consumption, and help build the ecological balance of nature.

### 2.3. Corporate Performance

Enterprise performance is the internal consideration and evaluation of the enterprise, which is expressed by relying on the financial indicators in the audit. The corporate social performance is a more comprehensive assessment, indicating the relationship between the organization and various stakeholders [23]. The basic framework of enterprise performance evaluation is shown in Figure 5.

From Figure 5, we can get the information that the sustainable development enterprise performance evaluation system is a “triple performance” evaluation model. It consists of three parts, namely economic performance, environmental performance, and social performance [24]. These three parts can be regarded as the three legs in its evaluation system, which stably support the evaluation system, and the relationship between these three legs is also very clear. In fact, the content of the enterprise performance evaluation system of sustainable development is the concept of sustainable development, stakeholders, and corporate social responsibility. These three subjects represent the evaluation indicators well. Because the main body of stakeholders has become more and more, the interests requested by everyone have also become different. The scope of performance evaluation is no longer limited to corporate economics but also adds corporate social responsibility and responsibility for protecting the environment. These three dimensions represent the sustainable development of enterprises [25].

The enterprise performance map can be seen in Figure 6 for details.

From Figure 6, we can know the information because green innovation and corporate responsibility are very closely related, and the behavior of enterprises not only affects the enterprise itself but also affects the whole society. Social performance is the external social responsibility image of an enterprise [26]. Enterprises should not only focus on making profits but should undertake social responsibilities. While it creates social wealth, it should also undertake corporate social responsibility. At the same time, the social performance also includes the economic contribution of the enterprise to society, and the enterprise also has the goal of creating value for society. Enterprises can drive the increase in employment rate and contribute tax revenue, which are all part of their social responsibility. Economic performance refers to the internal profitability of an enterprise, and the primary purpose of any enterprise is to strive for profits. If the goal of an enterprise is not to make profits, then the enterprise can only go into decline in the end. Its evaluation standard is mainly determined according to resource allocation and resource utilization, but it is very difficult to take into account both situations when evaluating. Therefore, the general evaluation will be carried out after different standards are formulated. The environmental benefit is an evaluation index extended according to the sustainable development of enterprises. In order to meet the needs of the current low-carbon society, environmental performance is added to the performance evaluation of enterprises. It mainly considers environmental performance. This assesses the company's environmental policy for the environment, the environmental goals achieved, and the environmental targets set. These environmental outcomes were measured [27].

### 2.4. SBM-DEA Model

This model is actually an efficiency evaluation method. Generally used in microeconomy, it can enrich theory and technology and can also reduce subjective factors and experimental errors and simplify algorithms [28]. However, because the traditional model has the problem of slack, the results will be unrealistic. In order to solve this problem, the SBM-DEA model was proposed.

*δ* is a non-negative number; then the decision-making unit can be expressed as follows:

(1) $$\begin{array}{c} C_{P}=\delta C+D^{-},\\ U_{P}=\delta U+D^{+}, \end{array}$$

where *D*^−^ is the input index and *D*^+^ is the output index; then the efficiency model of the slack index system can be expressed as follows:

(2) $$\begin{array}{c} YR_{P}=\text{MIN}\frac{1-1/N\sum_{O-1}^{N}D_{O}^{-}/C_{OP}}{1+1/D\sum_{O-1}^{D}D_{O}^{+}/U_{OP}},\\ \overset{M}{\underset{K=1}{\sum }}\gamma_{K}C_{U}+D_{K}^{-}=C_{OP},\\ \overset{M}{\underset{K=1}{\sum }}\gamma_{K}U_{OP}+D_{K}^{-}=U_{OP},\\ \overset{M}{\underset{K=1}{\sum }}\gamma_{K}=1.s. \end{array}$$

The linear programming is changed to get

(3) $$\begin{array}{c} YR_{P}=\text{MIN}Y\overset{M}{\underset{K=1}{\sum }}\frac{D_{O}^{-}}{C_{OP}},\\ \overset{M}{\underset{K=1}{\sum }}\gamma_{K}C_{U}+D_{K}^{-}=YC_{OP},\\ \overset{M}{\underset{K=1}{\sum }}\gamma_{K}U_{OP}+D_{O}^{+}=YU_{OP},\\ Y+\frac{1}{D}\overset{M}{\underset{K=1}{\sum }}\frac{D_{T}^{+}}{U_{TO}}=1,\\ \overset{N}{\underset{L=1}{\sum }}\beta_{L}=1. \end{array}$$

Output can be divided into desired output and undesired output. Then the sustainable innovation efficiency model can be constructed as follows:

(4) $$\begin{array}{c} P=\text{MIN}\frac{1-1/D\sum_{K=1}^{M}D_{T}^{+}/U_{TO}}{1+1/D_{1}+D_{2}\left(\sum_{K=1}^{M}D_{O}^{H}/C_{OP}^{H}+\sum_{K=1}^{M}D_{O}^{N}/U_{TP}^{N}\right)},\\ Y+\frac{1}{D_{1}+D_{2}}\left(\overset{M}{\underset{K=1}{\sum }}\frac{D_{O}^{H}}{C_{OP}^{H}}+\overset{M}{\underset{K=1}{\sum }}\frac{D_{O}^{N}}{U_{TP}^{N}}\right)=1. \end{array}$$

The CCR model is a more traditional model in DEA. If there are *M* units and *C*_*OP*_ represents the 0^th^ input index, it can get

(5) $$\begin{array}{c} YR_{P}=\text{MAX}\left(\frac{\sum_{T=1}^{D}I_{T}U_{TP}}{\sum_{O=1}^{N}B_{O}C_{OP}}\right). \end{array}$$

Transforming this formula, the following formula can be obtained:

(6) $$\begin{array}{c} YR_{P}=\text{MAX}\sum_{T=1}^{D}\beta_{T}U_{TP}. \end{array}$$

When *YR*_*P*_ is equal to 1, even transforming this formula, we can get

(7) $$\begin{array}{c} \text{MIN}\vartheta_{P}^{CCR}-\delta \left(\sum_{T=1}^{D}D_{O}^{+}+\sum_{T=1}^{N}D_{O}^{-}\right). \end{array}$$

## 3. Experiment and Green Innovation and Enterprise Sustainable Development Performance

### 3.1. Determination of Indicator Weights

The three indicators of corporate performance are listed above. Next, we will conduct a questionnaire survey to investigate the leaders and staff of an enterprise and ask them to evaluate the importance of indicators. Because they are very clear about the situation of the enterprise, their evaluation will be very realistic. The obtained results are shown in Table 1.

Information can be drawn from Table 1; the economic performance is divided into five parts. The profitability weight is 0.307. The weight of asset operating capability is 0.238. The weight for developing ability is 0.162. The weight of management capability is 0.063. The weight of innovation ability is 0.06. These are the results obtained by investigating the personnel of the enterprise. From the data in the table, we can know that the most important factor in economic performance is profitability because the primary goal of the enterprise is to make profits. Unprofitable businesses end up going out of business. The second is the asset operation capability because the enterprise needs asset coordination to operate. Then everyone thinks the least important is the ability to innovate. This is also in line with the current situation of most enterprises.

The weights of economic indicators are listed above, and the weights of social indicators are listed below, as shown in Table 2.

From the information in Table 2, the social performance indicators mainly have four parts. The weight of labor employment is 0.83. The weight of social influence is 0.127. The product liability weight is 0.556. The weight of human resources is 0.238. It can be seen that labor employment is the most important component of social performance because it bears the employment rate of most people. The second is product responsibility; the product designed by the company is to serve people. Therefore, if there is any problem with the product, the enterprise should be responsible for it. The least important is social impact, which may be compared to the fact that the people of the company feel that social impact is not enough part of social performance.

Then there are the weights of environmental performance indicators, as shown in Table 3.

From the information in Table 3, the EPI has three components. The weight of resource utilization is 0.62. It is the highest among the three parts, indicating that the strikes believe that resource utilization is the most important component of environmental performance. The requirement of a low-carbon society is to reduce the use of resources. The weight of emissions is 0.285, which is also considered important. Because the large amount of emissions produced by enterprises in the production process has caused adverse effects on the environment, emissions also occupy a place in environmental performance. The weight of environmental governance is 0.097. Because the first two parts are done, this part is not so important. Therefore, the company believes that the importance of environmental governance is relatively low.

### 3.2. Experiments Based on the SBM-DEA Model

In order to verify the reliability of the model in this paper, we collected the input-output data of a certain enterprise, as shown in Figure 7.

The information can be obtained from Figure 7. From 2017 to 2020, the fixed asset index of the company has always belonged to an upward trend, increasing year by year. The company's total profit is not very stable. This can be affected in many ways. But, overall, there is still an upward trend. The fixed asset value of the company in 2017 was 2,614,917.9; in 2018, it was 2,805,940.93; in 2019, it was 3,000,537.36; and in 2020, it was 3,765,123.2. The growth rate is still very fast, and it is expected to grow in the future, which shows that the fixed asset value of the company is very stable. The total profit of the company in 2017 was 81,835.5; in 2018, it was 244,419.8; in 2019, it was 159,091.83; and in 2020, it was 218,245.62. During this period, the total profit showed a loss, which shows that the production and operation of the enterprise were affected by other factors, but the overall profit curve still showed an upward trend.

In order to prove the excellent performance of the model, one enterprise may be less as a case, and we analyze the data of three enterprises. The enterprise performance efficiency excluding undesired outputs and the environmental efficiency of undesired outputs are compared. The result is shown in Figure 8.

From Figure 8, we can get the information that the performance efficiency of company A is the best. In the past 4 years, this enterprise has been at the forefront of efficient production, indicating that the input and output of this enterprise are very effective. Even in the case of sustainable development and green innovation, its efficiency is still at a high level. All aspects of the enterprise are developing in a balanced manner. In 2017, the efficiency of company A without unexpected output was 0.6943. The efficiency with undesired output is 0.6643. In 2018, the efficiency of the enterprise without undesired output is 1, and the efficiency with undesired output is 1. In 2019, the efficiency of the company without undesired output is 1, and the efficiency with undesired output is 1. In 2020, the efficiency of the company without undesired output is 1, and the efficiency with undesired output is 1. This shows that the company's performance in sustainable development is very good under green innovation. This also proves the applicability of the model in this paper from the side, using the efficiency of expected output and undesired output to compare, making the results more clear and specific.

Next, we make statistics on the Malmquist indices of the three companies without expected output, as shown in Figure 9.

From Figure 9, it can be seen that the Malmquist index of the latter two firms is greater than 1. In recent years, there have been great improvements in management and technology, and enterprises are also developing in a direction that is conducive to enterprise progress. A company's Malmquist index is between 0.9 and 1, which means that it has not developed comprehensively in terms of technical efficiency or technological progress. Its technical efficiency index is greater than 1, while the technological progress index is less than 1. Since the degree of impact of technological progress is greater than that of changes in technical efficiency, its Malmquist exponent is less than 1. That is to say, although the enterprise may have made some progress in enterprise management in a few years. But the extent of its lack of technical aspects hinders the production development of the entire enterprise. If all indexes of the enterprise are less than 1, the enterprise needs to adjust the strategic management structure to help the enterprise develop better. Without considering the undesired output, only company *B* is on the frontier, the performance efficiency of company A is relatively high, greater than 0.8, and the efficiency value of company *B* with relatively low efficiency is less than 0.4. Through the model listed in this paper, these data and information are well obtained, which shows that the model in this paper is very suitable for the analysis of enterprise sustainable development performance.

Below, we also conduct statistics on the Malmquist index of each company with the expected output, and the results are shown in Figure 10.

From Figure 10, it can be seen that the Malmquist index of firms A and B is greater than 1, and only the technical efficiency of the three firms is greater than 1. This shows that the management and technology of these two enterprises have been greatly improved in recent years, and the level of performance efficiency has a trend of developing in a good direction. The Malmquist index of enterprise A is between 0.9 and 1, which means that the development of production efficiency of this enterprise is uneven. The reasons are all a matter of technological innovation and change. In terms of efficiency, compared with the data without undesired output, the efficiency value of enterprises with undesired output has decreased to varying degrees. The average efficiency of the three companies is only 0.47, and the efficiency values of companies B and C are far lower than the average efficiency value. This shows that after taking into account the undesired output, the negative effect of this indicator has resulted in different degrees of impairment in comprehensive technology. This also means that firm efficiency evaluations that do not take into account the impact of undesired outputs are unrealistic. It further proves that the model in this paper can avoid the result distortion caused by the limitation of angle and radial direction of the traditional DEA model. It reflects the real enterprise performance efficiency and provides scientific and reliable data support for performance auditing.

## 4. Conclusion

This paper studies and analyzes the performance of green innovation and enterprise sustainable development through the SBM-DEA model and concludes that nonapplication of the model is of great help to the study of enterprise performance. It is more accurate and more realistic than the general model, making the output data more scientific and accurate. Therefore, further research on the implementation effect of this model can be considered. Due to the limited length of the article, it cannot cover all aspects, and there are not many examples used in the research. This is also the limitation of this paper. In the future, the author looks forward to using more real data to conduct in-depth research, so as to explore more methods for researching green innovation and corporate sustainable development performance. At the same time, we also firmly believe that there will be more and more researches on this topic in the future, and the sustainable development performance of enterprises will be better and better.

## Figures and Tables

**Figure 1:** Contents of green innovation.

**Figure 2:** Green innovation indicators.

**Figure 3:** Basic principles.

**Figure 4:** Connotation of sustainable development.

**Figure 5:** Basic framework.

**Figure 6:** Enterprise performance graph.

**Figure 7:** Input-output data: (a) value of fixed assets and (b) total profit.

**Figure 8:** Comparison of enterprise performance efficiency: (a) does not contain undesired outputs and (b) contains undesired outputs.

**Figure 9:** Statistics of Malmquist indicators of various enterprises without expected output.

**Figure 10:** Malmquist index statistics for companies with unexpected outputs.

**Table 1:** Economic indicators.

Index	Profitability	Asset operation	Development ability	Management ability	Creativity	Weights
Profitability	2	1/3	3	6	6	0.307
Financing	3	2	2	5	3	0.238
Development	1/5	2	2	4	4	0.162
Management	1/3	1/5	1/4	5	5	0.063
Innovation	1/3	1/5	1/4	1/3	1	0.060

**Table 2:** Social indicators.

Indicators	Labor and employment	Social influence	Product liability	The human resources	The weight
Indicators	2	1/3	1/5	1/4	0.83
Social influence	3	2	1/5	1/5	0.127
Product liability	6	5	2	5	0.556
The human resources	4	4	1/5	2	0.238

**Table 3:** Environmental indicators.

Indicators	Resource utilization	Emissions	Environmental governance	The weight
Resource utilization	2	4	5	0.62
Emissions	1/4	2	5	0.285
Environmental governance	1/5	1/5	2	0.097

## Data Availability

No data were used to support this study.
